This article has been retracted.

# Analysis of Intestinal Flora and Levels of Epidermal Growth Factor Receptor, Interleukin-32, and Gastrin 17 in Patients with Gastric Cancer via Carbon Nanoparticle Laparoscopy

**DOI:** 10.1155/2021/6697597

**Published:** 2021-05-12

**Authors:** Liping Bai, Fubing Yu, Lixian Bai, Yinhui Zhang, Zhi Li, Peng Li, Xueyan Yang, Zhijian Ma

**Affiliations:** ^1^Department of Gastroenterology, The Second People's Hospital of Yunnan Province, Kunming, 650021 Yunnan Province, China; ^2^Department of Neonatology, People's Hospital of Yuxi City, Yuxi, 653310 Yunnan Province, China; ^3^Department of Electronic Engineering, School of Information, Yunnan University, Kunming, 650021 Yunnan Province, China; ^4^Emergency Medicine Center, The First Hospital of Kunming, Kunming, 650021 Yunnan Province, China

## Abstract

In order to explore the changes of intestinal flora and serum levels of relevant substances in patients with gastric cancer before and after surgery with carbon nanoparticle laparoscopy, a total of 180 patients with early distal gastric cancer who adopted laparoscopic radical gastrectomy for distal gastric cancer in the general surgery department of TCM Hospital of Shi Jia Zhuang City from January 2018 to January 2020 were selected and randomly divided into two groups: traditional laparoscopic operation (control group) and carbon nanoparticle laparoscopic operation (experimental group) were adopted for treatment for the two groups, respectively. Postoperative evaluation included the difference between the two groups in the operative time, the efficiency of intraoperative lymph node dissection, and the number of lymph node detection. The adverse reactions, changes of intestinal flora before and after surgery in the two groups, and the serum levels of epidermal growth factor receptor (EGFR), interleukin-32 (IL-32), and gastrin 17 were evaluated. In the experimental group, the success rate of carbon nanoparticle tracer black staining reached 100%, and the operation time of the experimental group was significantly shorter than that of the control group (*P* < 0.05). The lymph node detection rate of the experimental group was higher than that of the control group (*P* < 0.05), but there was no significant difference in the lymph node metastasis rate between the two groups (*P* > 0.05). The sentinel lymph node sensitivity of the experimental group reached 92.3%, and the specificity, accuracy, and positive and negative prediction rates reached 100%; the experimental group patients were with an obviously higher incidence of level I-II gastrointestinal reaction (*P* < 0.05). Postoperative increases in Bifidobacteria and Lactobacillus were observed in both groups, while decreases in Enterococcus and Escherichia coli were observed in both groups (*P* < 0.05). Moreover, the degree of increase and decrease in the experimental group was greater than that in the control group (*P* < 0.05). The serum levels of EGFR, IL-32, and gastrin 17 in the two groups were significantly lower than those in the control group on 3 d, 7 d, and 15 d after surgery (*P* < 0.05). In the radical gastrectomy for distal gastric cancer, carbon nanoparticle laparoscopy was not only helpful for the localization of small tumors but also for the thorough dissection of lymph nodes after the surgery, and the postoperative adverse reactions of carbon nanoparticle laparoscopy were also less, which was of great significance for the improvement of intestinal flora and the reduction of serum levels of EGFR, IL-32, and gastrin 17 in gastric cancer patients.

## 1. Introduction

Gastric cancer is one of the four most common malignant tumors in the world, and its fatality rate ranks the top seven. It can be seen in the gastric antrum, the greater and lesser curvature of the stomach, and the anterior and posterior walls. China is a region with a high incidence of gastric cancer. According to the gastric cancer data report in 2015, there are estimated to be nearly 700,000 new cases of gastric cancer in China every year, and the mortality rate is about 500,000, ranking the second in both the incidence and mortality of malignant tumors [1]. According to statistical data, the incidence of gastric cancer in China is still at the highest [2]. At present, the clinical diagnosis of gastric cancer mainly relies on gastric cancer and pathological sections, but the patients' acceptability is poor, so it cannot be included in routine physical examination [3]. Most gastric cancer is originated from the mucosal epithelium of the stomach and belongs to adenocarcinoma, with an incidence in any part of the stomach and individualized symptoms, so misdiagnosis or missed diagnosis is very possible [4]. Lymph node metastasis is the most important prognostic indicator for both early and advanced gastric cancer. The lymph node metastasis rate in advanced gastric cancer can be as high as 70%, and even in early gastric cancer, the lymph node metastasis rate is around 20% [5, 6]. At present, the main imaging methods for gastric cancer include barium meal contrast examination, endoscopic ultrasound (EUS), computed tomography (CT), magnetic resonance imaging (MRI), and positron emission computed tomography-CT (PET-CT). Dual-energy CT and imaging omics have also been used in clinical studies. Barium meal radiography can directly observe the changes of gastric mucosa, lesion range, but cannot reflect the depth of lesion invasion, surrounding lymph nodes, and other organs involved. EUS combines the advantages of gastroscopy and ultrasound, which can simultaneously observe the surrounding lymph nodes and adjacent organs, but cannot detect the distant lymph nodes. MRI has high resolution but cannot be used as a routine examination. Laparoscopic radical surgery is a commonly used method for the treatment of gastric cancer. Compared with traditional abdominal root surgery, laparoscopic radical surgery can reduce the amount of blood loss and surgical trauma, which is conducive to postoperative recovery of patients. In recent years, due to the ideal delivery of various substances in the body and the tunable surface chemical targeting structure of various nanoparticles, laparoscopic radical surgery can show unique advantages in the targeted therapy of gastrointestinal diseases [7]. For patients with early gastric cancer, it can perform radical gastrectomy I, which can effectively remove the first group of lymph nodes around the stomach. For patients with advanced gastric cancer, radical gastrectomy type II can be performed, which can completely remove the second group of lymph nodes. For gastric cancer patients with lymph node metastasis in group 3, radical gastrectomy III should be adopted, which can completely remove lymph node metastasis in group 3 and obtain the best therapeutic effect.

Earlier studies on gastric cancer patients found that the intestinal flora of gastric cancer patients was significantly different from that of the healthy people, and the serum levels of EGFR, IL-32, and gastrin 17 were also significantly different from that of the healthy people [8]. Platinum is a common chemotherapy drug for gastric cancer, which has a high rate of adverse reactions in the digestive tract. Common clinical symptoms include nausea, abdominal distension, constipation, and diarrhea, which significantly affect the quality of life of patients [9]. In recent years, it was suggested that the adverse reactions of the digestive tract caused by chemotherapy were closely related to the maladjusted intestinal flora. Nanocarbon is a kind of lymph tracer widely used in clinic, which can negatively stain the parathyroid gland, and has the advantages of fast tracer speed and strong lymph tendency. Some researchers adopted carbon nanotracers to treat thyroid cancer. Nanocarbon tracer technology is accurate and simple for the identification of lymph nodes, which reduces the influence of human factors, improves the identification rate of lymph nodes, and effectively distinguishes the parathyroid gland, thus protecting it. Carbon nanotracers have a high degree of lymphatic tendency and specificity. In the treatment process of patients with gastric cancer, the adoption of carbon nanotracer technology to understand the status of intestinal flora plays an important role in the analysis and discussion of intestinal flora in patients with gastric cancer.

IL-23, an important component of inflammatory cytokines, has been shown in many studies to have proinflammatory properties. However, few studies observed the expression of IL-23 in gastric cancer. Gastrin 17 is secreted by gastric antrum cells and is a noninvasive biological indicator of the structural and functional state of the gastric mucosa. It was reported that gastrin 17 promoted the regeneration and replication of pancreatic beta cells and stimulated insulin secretion. Sustainably high levels of gastrin 17 suggest irreversible lesions, so evaluating gastrin 17 helps to determine clinical efficacy.

Based on the above problems, the nanocarbon tracer technology was innovatively combined with intestinal flora status and serum levels of EGFR, IL-32, and gastrin 17 in gastric cancer patients in this study. The clinical effects of carbon nanoparticle tracer technology could be explored by evaluating the above indicators, so as to guide the clinical application of nanocarbon tracer and provide a reliable basis for the localization of sentinel lymph node of gastric cancer by nanocarbon tracer staining and the determination of lymph node metastasis.

## 2. Materials and Methods

### 2.1. Study Objects and Grouping

A total of 180 patients with early distal gastric cancer who adopted laparoscopic radical gastrectomy for distal gastric cancer in the general surgery department of TCM Hospital of Shi Jia Zhuang City from January 2018 to January 2020 were selected as study objects. All patients were diagnosed with early distal gastric cancer by more than two physicians. 180 patients were randomly divided into two groups with 90 patients in each group. There were 48 males and 42 females in the experimental group, with an average age of 51.26 ± 5.08. There were 53 males and 37 females in the control group, and the average age was 52.17 ± 4.85 years. There was no significant difference between the two groups in age, gender, degree of gastric cancer, and extent of invasion (*P* > 0.05).

All the 90 patients in the experimental group were labelled with carbon nanoparticle lymphoid tracer before operation, and no patient was converted to open laparotomy, and there were no adverse drug reactions or other complications at the injection site. Patients in the control group were not labelled with a carbon nanoparticle lymphoid tracer before operation, and no patient was converted to open laparotomy. All patients evolved in the experiment had signed informed consent forms, and this study was reviewed and approved by the hospital ethics committee.

### 2.2. Inclusion Criteria and Exclusion Criteria

The inclusion criteria of patients participating in the experiment were as follows: (I) gastric cancer was confirmed by electronic gastroscopy and pathological diagnosis on admission, and the cancer tissues were only limited to the mucosal layer or submucosa by clinical endoscopic ultrasonography; (II) the patient's lesion was a single lesion, without metastasis or tumor in other sites; (III) chest and abdomen metastasis was detected by preoperative chest and abdomen combined with enhanced CT; (IV) MRI scan around the tumor showed no infiltration of surrounding tissues and organs. Exclusion criteria were as follows: (I) patients in pregnancy and early pregnancy; (II) patients with severe cardiovascular and cerebrovascular diseases, liver and kidney diseases, and hematopoietic dysfunction; (III) those whose expected survival period did not exceed 6 months; (IV) patients with a history of tumor; (V) patients adopted major abdominal operation or had a history of abdominal trauma; (VI) adjuvant chemoradiotherapy was performed before operation; (VII) patients with cerebral infarction, cerebral hemorrhage, or other brain diseases; (VIII) patients who had already participated in other clinical trials.

### 2.3. Preoperative Staining and Operation Methods

Preoperative staining was as follows. The experimental group was stained with carbon nanoparticle tracer 24 h before operation, which was manufactured by Chongqing Laimei Pharmaceutical Co. Ltd., and named as carnaline. The injection was performed at 4-5 sites around the gastric mucosa surrounding the tumor observed by electronic gastroscopy 24 hours before operation. When the injection needle penetrated into the submucosa and slowly pushes about 5 mm, the injection was carried out, and the injection volume of each site was 0.15~0.2 mL. Before the needle was pulled out, a certain amount of nanotracer was pumped back to prevent exosmosis of carbon nanoparticles.

Operation methods: both groups were operated by the same surgical team skilled in laparoscopic radical gastrectomy for distal gastric cancer. The same operation was performed in both groups, and the specific operation was as follows. The patient was in a “herringbone” position on the operating table and adopted general anaesthesia with endotracheal intubation. The minimally invasive laparoscopic operation was performed with a 5-hole method. An observation hole was opened about 1 cm below the umbilicus, and a 30-degree laparoscopic lens was used for observation. Four puncture holes were made in the left and right abdomens, respectively, for operation holes and auxiliary operation holes. During the operation, the carbon dioxide pneumoperitoneum was established and the pressure of the pneumoperitoneum was set at 12 mmHg. Then, the abdominal and pelvic cavity was examined to confirm the specific location of the tumor and the presence of metastasis. A series of procedures were then performed, including intraoperative noncontact separation of the tumor, complete resection of the tumor, and protection of the gastric wall incisions near and far of the tumor. The scope of intraoperative lymph node dissection included D1 lymph node dissection (including lymph node dissection in group 1, group 3, group 4sb, group 4d, group 5, group 6, and group 7). Lymph node dissection was performed in group 8a, group 9, group 11p, and group 12a.

### 2.4. Lymph Node Counting and the Definition of the Sentinel Lymph Node

The black staining of lymph nodes was observed intraoperatively by laparoscopy, and the total operative time of patients in both groups was recorded after thorough lymph node dissection at stage 2. Lymph nodes were screened, classified, and counted in vitro by an attending physician with a certain number of years of experience. The count of the experimental group was as follows. The lymph nodes with black staining and closest to the gastric tumor in the experimental group were defined as sentinel lymph nodes, which were separately collected and bagged for storage. All lymph nodes with black staining were counted and grouped, and finally, the lymph nodes with black staining that could be touched were selected by naked eye and touch. In the control group, the count was as follows. All lymph nodes were detected as far as possible directly by naked eye and touch.

### 2.5. Postoperative Adverse Reaction Index Standard

Postoperative adverse reactions of the two groups were evaluated, respectively. To make the evaluation easier, adverse reactions were classified as follows: proteinuria: level I: <0.3 g/100 mL, level II: 0.3 ~ 1.0 g/100 mL, level III: >1.0 g/100 mL, and level IV: nephrotic syndrome; hypertension: level I: 140/90~159/99 mmHg, level II: 160/100~179/109 mmHg, level III: >179/109 mmHg, and level IV: high pressure; leukopenia: level I: (3.0 ~ 3.9) × 10^9^/L, level II: (2.0 ~ 2.9) × 10^9^/L, level III: (1.0 ~ 1.9) × 10^9^/L, and level IV: <1.0 × 10^9^/L; hemorrhage: level I: petechiae, level II: mild blood loss, level III: significant blood loss, and level IV: severe blood loss; skin of hands and feet: level I: erythema, level II: dry desquamate and blister, level III: wet dermatitis and ulcer, and level IV: exfoliative dermatitis and necrosis; gastrointestinal reaction: level I: nausea and transient abdominal pain and diarrhea, level II: temporary nausea or tolerable abdominal pain and diarrhea, level III: vomiting or diarrhea due to unbearable abdominal pain, and level IV: uncontrollable vomiting or bloody diarrhea.

### 2.6. Intestinal Flora Collection and Serum-Related Substance Collection and Detection

Before and after surgery, 3-5 g stool samples were collected and placed in sterile vials. According to the different environment required by the growth of bacteria, the appropriate culture medium was selected successively for culture. The bacteria were cultured in an incubator at 37°C, and the bacterial content in the cultured fecal diluent was calculated successively. The counted bacteria included Bifidobacteria, Lactobacillus, Enterococcus, and Escherichia coli. The bacteria content in each gram of feces was expressed in the form of log10n. Fasting blood 2 mL of abdominal and elbow venous blood was extracted from patients of the two groups from the morning of 3 d, 7 d, and 15 d before and after surgery, respectively. Centrifugation was performed at 3000 rpm for 10 min, and then, the upper serum was removed. Serum levels of EGFR, IL-32, and gastrin 17 were detected by enzyme-linked immunosorbent assay (ELISA) (BD, USA).

### 2.7. Statistical Analysis

SPSS 19.0 software was adopted for statistical analysis. The counting results were expressed as mean plus or minus standard deviation $\left(\bar{x}\pm s\right)$, *t*-test was adopted for comparison between the two groups, and the chi-square test was used for count data. *P* < 0.05 was considered statistically significant.

## 3. Results

### 3.1. Comparison of General Data of Patients

The comparison results of general data between the experimental group and the control group are shown in Figure 1. The age, gender, tumor site, and tumor differentiation degree of the two groups were compared, and the difference between the two groups was not statistically significant (*P* < 0.05).

### 3.2. Operation Results

90 patients in the experimental group and 90 patients in the control group were successfully performed and completed laparoscopic operation as planned, and all the patients were not converted to laparotomy during the operation. No adverse reactions or suspected adverse reactions were found in the experimental group. In the experimental group, due to the administration of carbon nanoparticle lymphoid tracer, significant lymph nodes were observed to be blacken around the gastric cancer under high-definition laparoscopic observation, and there was no black staining in the surrounding retinal tissue and adipose tissue, so the carbon nanoparticle tracer would not hinder the operation and the doctor's determination of the anatomical level, as shown in Figure 2.

All 180 patients in the experimental group and the control group were successfully operated, that was, lymph nodes of gastric cancer patients in the experimental group achieved 100% success through black staining of carbon nanoparticle tracer technology. Compared with the control group, the operation time of the experimental group was significantly shortened, and the difference was statistically significant (*P* < 0.05), as shown in Figure 3.

### 3.3. Overall Lymph Node Detection Results

The average number of lymph nodes detected in the experimental group was 32.4 ± 7.3, while the average number of lymph nodes detected in the control group was 19.61 ± 6.23, the number of lymph nodes in the experimental group was larger than that in the control group, and the difference was statistically significant (*P* < 0.05). Small lymph nodes (diameter less than 5 mm) detected in the experimental group accounted for 60.8% of the total, and those detected in the control group accounted for 43.27%. The number of lymph nodes in the experimental group was larger than that in the control group, and the difference was statistically significant (*P* < 0.05). The lymph node metastasis rate was 16.2% in the experimental group and 15.7% in the control group, and the difference was not statistically significant (*P* > 0.05), as shown in Figure 4.

### 3.4. Sentinel Lymph Node Detection and Metastasis

In all 90 patients of the experimental group, the carbon nanoparticle tracer successfully located the sentinel lymph nodes, and the detection success rate reached 100%. Meanwhile, pathological results showed that 13 patients were confirmed to have regional lymph node metastasis, including 12 patients with positive sentinel lymph node; among the 13 patients with lymph node metastasis, 46 lymph nodes with metastasis were detected; and a total of 41 metastatic lymph nodes were detected in 12 patients with a positive sentinel lymph node. Based on the above results, the sensitivity, specificity, accuracy, positive prediction rate, and negative prediction rate of carbon nanoparticle tracer for tracing sentinel lymph node could reach 92.3%, 100%, 100%, 100%, and 100%, respectively.

### 3.5. Comparison of Postoperative Adverse Reactions

Compared with the control group, the experimental group patients were with an obviously higher incidence of level I-II gastrointestinal reaction (*P* < 0.05), and the proteinuria, hypertension, leukopenia, bleeding, skin reactions of hands and feet, and the incidence of gastrointestinal reaction of level III-IV were not statistically significant (*P* > 0.05), as shown in Figure 5.

### 3.6. Comparison of Intestinal Flora Content

Before the operation, the contents of Bifidobacteria, Lactobacillus, Enterococcus, and Escherichia coli in the intestines of the two groups were not statistically significant (*P* > 0.05). After the operation, the contents of Bifidobacteria and Lactobacillus in both groups increased significantly, while the number of Enterococcus and Escherichia coli decreased significantly, and the difference was statistically significant (*P* < 0.05). The increased amplitude of Bifidobacteria and Lactobacillus and the decreased amplitude of Enterococcus and Escherichia coli in the experimental group were significantly larger than those in the control group, and the difference was statistically significant (*P* < 0.05), as shown in Figure 6.

### 3.7. Comparison of Changes in Levels of EGFR, IL-32, and Gastrin 17

The serum levels of EGFR, IL-32, and gastrin 17 were not significantly different between the two groups before and after surgery (*P* > 0.05). At 3, 7, and 15 days after surgery, serum levels of EGFR, IL-32, and gastrin 17 in the two groups were significantly decreased, and the decrease in the experimental group was significantly greater than that in the control group, with statistically significant difference (*P* < 0.05), as shown in Figure 7.

## 4. Discussion

Gastric cancer is one of the most common cancer types in China. According to the statistical data of Cancer Report 2019 in China, the incidence and deaths of gastric cancer in China account for about half of the world's total [10]. At present, the treatment of gastric cancer mainly involves radical resection, which is also recognized as the best treatment for gastric cancer [11–13]. At present, laparoscopic mucosal resection is mostly used in clinical treatment, but a study of Khazaei et al. (2019) [14] showed that even under strict operation, the current laparoscopic surgery could not be guaranteed to be completely radical. As a standard operation for the treatment of early gastric cancer, D2 radical resection requires lymph node dissection in addition to the removal of 2/3 of the stomach. However, whether the dissection is performed and the scope of the dissection judged by the naked eye will cause gastric wall damage to the patient [15, 16].

Therefore, the carbon nanoparticle tracer was introduced to assist the confirmation of the cleaning range in this experiment. The experimental results showed that the operation time of patients using carbon nanoparticle tracer was significantly shorter than that of the control group, and the number of lymph nodes at the site of dissection was also significantly higher than that of the control group, which was the same as the results of animal experiments conducted by Arends et al. (2017) [17]. And it was found that the sensitivity of carbon nanoparticle tracer tracing to sentinel lymph node to evaluate regional lymph node metastasis could reach 92.3%, and the specificity, accuracy, positive prediction rate, and negative prediction rate were all up to 100%. This experimental result further verified the feasibility of using sentinel lymphocytes to predict metastasis shown in a study of Ralls et al. (2016) [18]. The postoperative adverse reactions of patients conducting operation using carbon nanoparticle tracer were significantly lower than those in the control group, which may be related to the fact that carbon nanoparticle tracer could accurately mark the dissection range, so as to avoid excessive dissection. A study of Wang et al. (2018) [19] showed that extensive lymph node dissection in gastric cancer patients would greatly increase postoperative adverse reactions, and intestinal flora and serum levels of EGFR, IL-32, and gastrin 17 in the experimental group were also improved, which was largely related to the degree of lymph node dissection. The animal experiments of Wang et al. (2017) [20] also showed that the degree of lymph node dissection in animals with gastric cancer was associated with the recurrence of gastric cancer.

## 5. Conclusion

In this study, whether the regional lymph nodes were metastatic lymph nodes was evaluated through the carbon nanoparticle tracer in early laparoscopic distal operation and their blackening status. In this study, the success rate of carbon nanoparticle tracer laparoscopy was 100%, the operation time was significantly shorter than that of the control group, and the lymph node dissection was more thorough. The adverse reactions, intestinal flora, and serum levels of EGFR, IL-32, and gastrin 17 in the two groups were compared and evaluated before and after the operation; it was found that the postoperative adverse reactions were more obvious in the control group than those in the experimental group. Compared with those before operation, intestinal Bifidobacteria and Lactobacillus increased while Enterococcus and Escherichia coli decreased in both groups, and the degree of increase and decrease in the experimental group was greater than that in the control group. The serum levels of EGFR, IL-32, and gastrin 17 in the two groups were decreased compared with those in the control group, and the reduction in the experimental group was greater than that in the control group. The results of this study showed that carbon nanoparticle tracer laparoscopy had a better therapeutic effect and lower postoperative adverse reaction rate, and the structure of intestinal flora and serum levels of EGFR, IL-32, and gastrin 17 could be changed more effectively. However, the realization of carbon nanoparticle tracer laparoscopy required the cooperation of all departments in hospitals, and more clinical trials were needed to achieve the true clinical application.

## Figures and Tables

**Figure 1:** Comparisons of general data of patients.

**Figure 2:** Laparoscopic image after carbon nanoparticle lymphoid tracer injection.

**Figure 3:** Comparison of operation time.

**Figure 4:** Overall lymph node detection results: (a) average number of lymph nodes, (b) proportion of small lymph nodes, and (c) lymph node metastasis rate.

**Figure 5:** Comparison of adverse reactions between the two groups.

**Figure 6:** Comparison of intestinal flora content between the two groups before and after surgery: (a) control group and (b) experimental group.

**Figure 7:** Changes of serum levels of related substances in both groups before and after surgery: (a) EGFR, (b) IL-32, and (c) gastrin 17.

## Data Availability

Some or all data, models, or codes generated or used during the study are available from the corresponding author by request.
